# Investigation of Applying Machine Learning and Hyperparameter Tuned Deep Learning Approaches for Arrhythmia Detection in ECG Images

**DOI:** 10.1155/2022/8571970

**Published:** 2022-09-12

**Authors:** Kogilavani Shanmugavadivel, V. E. Sathishkumar, M. Sandeep Kumar, V. Maheshwari, J. Prabhu, Shaikh Muhammad Allayear

**Affiliations:** ^1^Department of Computer Science Engineering, Kongu Engineering College, Perundurai, Erode, 638 060 Tamil Nadu, India; ^2^Department of Industrial Engineering, Hanyang University, Seoul, Republic of Korea; ^3^School of Information Technology and Engineering, Vellore Institute of Technology, Vellore, 632014 Tamil Nadu, India; ^4^Department of Multimedia and Creative Technology, Daffodil International University, Daffodil Smart City, Khagan, Ashulia, Dhaka, Bangladesh

## Abstract

The level of patient's illness is determined by diagnosing the problem through different methods like physically examining patients, lab test data, and history of patient and by experience. To treat the patient, proper diagnosis is very much important. Arrhythmias are irregular variations in normal heart rhythm, and detecting them manually takes a long time and relies on clinical skill. Currently machine learning and deep learning models are used to automate the diagnosis by capturing unseen patterns from datasets. This research work concentrates on data expansion using augmentation technique which increases the dataset size by generating different images. The proposed system develops a medical diagnosis system which can be used to classify arrhythmia into different categories. Initially, machine learning techniques like Support Vector Machine (SVM), Naïve Bayes (NB), and Logistic Regression (LR) are used for diagnosis. In general deep learning models are used to extract high level features and to provide improved performance over machine learning algorithms. In order to achieve this, the proposed system utilizes a deep learning algorithm known as Convolutional Neural Network-baseline model for arrhythmia detection. The proposed system also adopts a novel hyperparameter tuned CNN model to acquire optimal combination of parameters that minimizes loss function and produces better result. The result shows that the hyper-tuned model outperforms other machine learning models and CNN baseline model for accurate classification of normal and other five different arrhythmia types.

## 1. Introduction

Humans find object classification to be a relatively simple operation, but machines have found it to be a difficult problem; hence, image classification has become a critical task. Image classification is the process of categorizing images into one of several predetermined categories. A single image can be classified into an endless number of categories [1]. Manually evaluating and classifying these images can be time-consuming, especially when there are a big number of them; therefore, automating the process using machine learning and deep learning techniques would be quite beneficial. Particularly, these algorithms are really helpful to get precise results in medical domain like COVID-19 detection [2]. According to the World Health Organization (WHO), Cardiovascular Disease (CVD) is the main reason for heart attack [3]. The World Heart Federation says that, by 2030, there may be more than 23 million CVD-related deaths per year. Any irregular abnormality from normal heart rhythms leads to a type of CVD disease known as arrhythmia. A succession of arrhythmia heartbeats can be harmful, even though a single pulse may not have a substantial influence on one's life. The proposed work applies CNN with electrocardiogram (ECG) grayscale images to create an effective arrhythmia classification method in order to classify ECG images into six categories, one being normal and the other five being distinct types of arrhythmia like Left Bundle Branch Block (LBBB), Right Bundle Branch Block (RBBB), Premature Atrial Contraction (PAC), Premature Ventricular Contraction (PVC), and Ventricular Fibrillation (VF). The contribution of this research work is as follows:

- A novel hyper-tuned CNN model is proposed for the detection of arrhythmia
- Data augmentation is performed generating a large dataset
- ECG grayscale images are collected from Kaggle, and UCI repository can be used as input
- Five different types of arrhythmia are detected by applying machine learning, CNN-Baseline model, and hyper-tuned model

Various solutions for high-class imbalance across data types are discussed in [4]. Recent reviews unveil that the accuracy of the learned models may be improved by data augmentation. Data warping-based image augmentation is used in LeNet-5 [5], and it is the first application in which CNN is applied for handwritten digit classification. In [6], dataset size is increased by augmentation by applying cropping, flipping, and changing the intensity using PCA. Image data augmentation is a technique for increasing the size of the dataset artificially by producing different images of the same dataset. This is a method of applying various transformations to original images in order to create many modified versions of the same image. Each duplicate, on the other hand, differs in various ways, based on the techniques applied such as shifting, rotating, and flipping. These transformed images are mainly used by the algorithms for classification.

A CNN-Transformer-based model is applied to detect three different arrhythmia types in [7], and the mentioned method is applied to MIT-BIH dataset. A clustering-based approach is adopted in [8] to predict four types of arrhythmia. In this work, statistical index based on phase-space analysis is carried out for both prediction and classification. In order to distinguish between healthy heartbeat and pathological rhythms, data analysis can be carried out on edge devices in [9] using deep CNN. Purely rhythm-based methodology is introduced in [10] by computing RR-interval sequences from ECG signals, and for arrhythmia classification, LSTM is utilized. In order to identify the origin of the focal arrhythmia wave front, prediction curves can be generated in [11]. The numbers of neurons, activation function, optimizer, learning rate, batch size, and epochs are all tuned via hyperparameters. Convolution neural networks are used in computer vision to develop models for image-related processes such as image categorization and object detection. A CNN model is formed by combining multiple convolution layers, pooling layers, dropouts, and finally fully linked layers in image classification applications. However, hyperparameters in the CNN model may be tuned in order to obtain best results.

The main findings of this research work are that in order to obtain better accuracy, the proposed system adopts data augmentation and novel hyper-tuned CNN model. We performed evaluation on five different types of arrhythmia types from the dataset collected from Kaggle and UCI repository. The ImageDataGenerator class in Keras library is used to produce augmented images. To determine the best parameters in the CNN hyper-tuned model, Keras Tuner library is used.

The organization of this research paper is presented here. The literature survey about arrhythmia detection is discussed in Section 2. The proposed methodology is explained in Section 3, and it also gives full description of classification models utilized.  Section 4 describes performance analysis of all the proposed models. Finally, in Section 5, the conclusion and future work are specified.

## 2. Literature Survey

The recent research work that can be carried out for ECG image classification by various learning approaches, dataset utilized, and results obtained is presented in Table 1.

The most frequently occurring problem when working with machine learning and Deep Neural Networks is that there is insufficient amount of training data or class imbalance among the dataset. One way to deal with this problem is data augmentation. In [27], the image style transfer method is proposed to perform various image transformations. Basic image transformations like color, geometric, and mixing of images are discussed in [28]. New samples were created from an existing dataset by performing translation and rotation as mentioned in [29].

## 3. Proposed System

The proposed system collects ECG image data from Kaggle and UCI repository [30, 31]. In order to get the variant of dataset, data augmentation is performed. Initially, training data is applied to state-of-the-art learning methods like SVM, Naïve Bayes, and Logistic Regression. In addition to that, an augmented dataset is applied to deep learning models like baseline CNN and CNN with hyper-tuned parameters. A trained model is validated using validation data and tested using unseen data. The proposed models classify ECG-based image dataset into normal as well as five different arrhythmia types or classes like LBBB, PAC, PVC, RBBB, and VF. The proposed system workflow is represented in Figure 1.

### 3.1. Dataset Description

The dataset utilized for this work is collected from Kaggle and UCI repository. The dataset contains six classes which includes normal rhythm with abnormal heart activity known as arrhythmias. The shapes of different types of arrhythmias that can be found in ECG images are shown in Figure 2.

### 3.2. Data Augmentation Techniques

Training datasets can be made larger and of higher quality by adding additional data. The ImageDataGenerator component of the Keras framework is used in the proposed system to apply various transformation functions to all of the original images at various epochs. The recently created images contain various iterations of the same image and are used in deep learning and machine learning techniques. At each epoch, Keras ImageDataGenerator class produces different images for analysis purpose. But these augmented images need not be included in the original dataset due to overfitting problem. Another benefit of ImageDataGenerator is that it consumes less memory. This is because if you did not utilize this class, all of the images would have loaded at the same time. However, when it is used, the images are loaded in batches, saving a lot of memory. Standardization, rotation, shifts, flips, brightness alteration, and many other augmentation techniques are available in Keras. Before any subsequent processing, the data is multiplied by a value called rescale. Shear range is used to apply shearing transformations at random. A dataset obtained after applying data augmentation techniques is described in Table 2.

ECG images can be rotated freely between 0 and 360 degrees by using an image rotation data augmentation technique. As the image is rotated, certain pixels will move outside the image, creating an empty space that needs to be filled in. This value can be filled in a variety of ways, such with a constant value or by nearest pixel values. To make the object to be at the centre of the ECG image, the pixels can be relocated either in a horizontal or vertical way. This can be done using height shift range and width shift range parameters. Flipping ECG images is another wonderful enhancement technique that can be applied to a variety of objects. The ImageDataGenerator class offers arguments like horizontal flip and vertical flip. This technique, however, should be used in accordance with the object in the ECG image. The random brightness of the ECG image is changed at random. It is also a highly effective augmentation approach. The brightness range option in the ImageDataGenerator class can be used to regulate the brightness. Values greater than 1.0 are used to brighten the ECG image. After applying the mentioned data augmentation techniques, sample ECG image is specified in Figure 3.

### 3.3. Machine Learning Models

A mathematical representation of the patterns concealed in data is represented through different machine learning models. When this model is trained on data, it develops some sort of controlling structure. This may be converted into rules that will be helpful for predicting new scenarios. So, if a model is trained on certain training data and then applied to fresh data, the model will be able to infer some sort of link. Various machine learning approaches, purpose, and advantages are discussed in [32]. Support Vector Machine is a supervised machine learning approach that may be applied to both regression and classification tasks. When used for classification, it uses a linear boundary to divide the classes. It creates a hyperplane or a series of hyperplanes and is used to create good separation between the two classes [33]. The kernel function that is employed determines the algorithm's true power. The Naive Bayes algorithm adopts the Bayes theorem and works under the assumption that attributes are unrelated. Even when other variables are available, it is impossible to know anything about other aspects [34]. So, the augmented dataset is applied to this algorithm to detect arrhythmia types without explicitly knowing about other parameters or attributes present in the dataset. Logistic regression is used to calculate the likelihood of a class [35]. The proposed system utilizes logistic regression to classify the given ECG images into five arrhythmia types.

### 3.4. Deep Learning Models

Deep learning is a subfield of machine learning that is becoming increasingly popular. Neural networks are used to create deep learning models. A neural network processes inputs by feeding them into hidden layers with weights that are adjusted during training. The model then issues a forecast. The weights are altered to discover patterns in order to produce better forecasts. Because the neural network learns on its own, the user does not need to define what patterns to look for. Keras is a Python-based neural network library that is easy to use. Each input image in a Convolutional Neural Network goes via two convolutional blocks, or two convolution layers, a pooling layer and a dropout layer for regularisation. Finally, each output is flattened and passed through a thick layer that sorts the image into one of six categories.

#### 3.4.1. CNN-Baseline Model

A Convolutional Neural Network is a special category of the Artificial Neural Network which accepts images as inputs. The sequential model is developed as a baseline model by adding the convolution layer with filters and activation function. Then, the max pooling layer, hidden layer, and output layer are added. Then, the model is compiled and trained and evaluated. While the design of the Neural Network is vital for extracting information from input, updated rules based on the gradient of the loss function are used to improve everything. The optimizer determines the updating rules. Adam is a well-known optimizer that is still in use in most neural networks. It uses an exponential declining average of the gradient, and it is squared to update the variables. The organization of CNN baseline model is shown in Figure 4.

The model type used in the CNN-Baseline model is sequential. During a model building process, multiple layers are added and ReLU is the activation function employed in the first two layers. Input shape is (64, 64, 1) with the value 1 indicating that the given images are in greyscale. A flatten layer is in between the Conv2D layers and the dense layer. It is used to connect the convolutional and dense layers. The output layer is dense, and it contains 6 nodes, one for each conceivable outcome (0–5). Softmax is the activation function to reduce the output to a single number. The CNN-Baseline model summary is specified in Table 3.

#### 3.4.2. CNN-Hyper-Tuned Model

There are so many hyperparameters in neural networks that manually tuning them is nearly impossible. Keras Tuner makes tuning the hyperparameters of neural networks a breeze. Deep learning model development is an iterative process in which you start with a basic architecture and then tweak it until you have a model that can be trained efficiently in terms of both time and computing resources. To achieve this, adjust the settings of hyperparameters, and repeat the process until get the good performance. Hyperparameter tuning is the process of identifying a good collection of hyperparameters. For more complicated models, the number of hyperparameters might skyrocket, and manually tweaking them can be difficult. To address this issue, the proposed system utilizes Keras tuner. It is a library for tweaking the hyperparameters of a neural network that aids in the selection of ideal hyperparameters in a TensorFlow neural network. The model that utilizes Keras tuner is called a hyper-tuned model because it fine tunes the hyperparameters. The workflow of hyperparameter tuning process is represented in Figure 5.

Randomly sampling hyperparameter combinations and testing them out is the most straightforward technique to undertake hyperparameter tweaking. First, choose an ideal value between 32 and 512 for the number of units in the first dense layer.

In order to specify the search space for dense units, minimum and maximum values, as well as the step size used to increment between them, are needed to be specified. Next, the optimizer's learning rate is adjusted by selecting an appropriate value from 0.01, 0.001, or 0.0001. During hyper tuning process, the selection of learning rate allows to designate discrete values to include in the search space. The process to be followed to obtain hyper tuned model is specified in Figure 6.

The tuner is then instantiated and the hyperparameters are tuned. The Hyper Band Tuner algorithm is used to optimize hyperparameters in this way. To swiftly converge on a high-performing model, it employs adaptive resource allocation and early-stopping. The number of models to run is determined by this procedure. The following step is to look for the best hyperparameter. Finally, create the model using suitable hyperparameters, and train it. The CNN-hyper tuned model summary is specified in Table 4.

## 4. Performance Evaluation

The precision score is a measure of how well the model predicted the positives out of all the positive predictions it generated. The accuracy score is a good predictor of prediction success when the classes are severely unbalanced. In mathematics, it displays the proportion of true positives to the total of true positives and false positives. By accurately calculating the number of true positives among all positive predictions, it is used to evaluate the model's performance. This value is calculated as mentioned in

(1) $$\begin{array}{c} \text{Precision}=\frac{\text{TP}}{\text{FP}+\text{TP}}. \end{array}$$

The recall score assesses the model's ability to accurately forecast positives from genuine positives. This is distinct from precision, which measures the proportion of accurate predictions a model makes among all accurate forecasts. It evaluates how effectively our machine learning model distinguishes between all genuine positives and all probable positives in a dataset. The recall score increases as the machine learning model becomes more adept at distinguishing between positive and negative data. Recall score is a good predictor of prediction success when the classes are severely unbalanced. In mathematics, it is the proportion of genuine positives to the total of true positives and false negatives. In terms of precisely counting true positives among all the real positive values, it is used to evaluate the model's performance. Recall value is calculated using

(2) $$\begin{array}{c} \text{Recall}=\frac{\text{TP}}{\text{FN}+\text{TP}}. \end{array}$$

The accuracy metric for machine learning models is the proportion of true positives and true negatives to all positive and negative observations. In other words, accuracy represents the probability that, given the total number of predictions our machine learning model being made, it would correctly predict a result. It is the ratio of all mathematically accurate positive and negative predictions. By computing the ratio of true positives to true negatives over all forecasts, it is used to evaluate the model's performance. Accuracy is calculated using

(3) $$\begin{array}{c} \text{Accuracy}=\frac{\text{TP}+\text{TN}}{\text{TP}+\text{FN}+\text{TN}+\text{FP}}. \end{array}$$

The F1-Score is a representation of the model score as a function of recall and precision. It is typically used as a single value that offers comprehensive information about the model's output quality. Mathematically, it can be written as the harmonic mean of the precision and recall score. When choosing either accuracy or recall score can lead to a model with significant false positives and false negatives, the F1-Score, which is the harmonic mean of the two scores, is employed as a statistic. It is calculated using

(4) $$\begin{array}{c} \text{F}1‐\text{Score}=\frac{2*P*R}{P+R}. \end{array}$$

The precision, recall, F1-Score, and accuracy for various machine learning algorithms and CNN algorithm baseline model and hyper-tuned model for validation dataset are shown in Table 5.

Optimizer, loss, and metrics are the three parameters used to build the model. The optimizer manages the learning rate. The CNN-Baseline model makes use of the Adam optimizer. Adam is a good optimizer to use, on the whole. For classification problems, the “categorical cross entropy” loss function is frequently employed. If the score is lower, the model is operating more effectively. Finally, the accuracy measure is utilized to determine the accuracy score on the validation set when we train the model. After each optimization iteration, a model's performance is shown by its loss value. Loss is defined as the difference between the problem's true values and the model's anticipated values. Model parameters are updated based on this loss value. A great accuracy with low loss means low errors on a dataset.

The precision, recall, F1-score, and accuracy values obtained by various machine learning models and deep learning models are shown in Figures 7–10. The result shows that with the help of hyperparameter tuning, the CNN-hyper-tuned model obtained the highest values compared to all other models.

Figure 11 shows accuracy and loss values of CNN-Baseline model for 20 epochs. The values show that training dataset loss is reduced from 1.0222 to 0.0889. Validation dataset loss is reduced from 0.8079 to 0.3438. Training dataset accuracy is improved from 0.6383 to 0.9724. Validation dataset accuracy is improved from 0.7163 to 0.9118 due to the fact that applying the CNN-Baseline model for 20 epochs in which each and every epoch the model automatically learn significant features from data.

Five different trials that output the trial summary and the best hyperparameters in the CNN-Hyper-tuned model are shown in Table 6. The result shows that at trail 4, the CNN-Hyper-tuned model obtained the best validation accuracy of 0.94375 using Random Search. With the help of Keras tuner, the proposed CNN-Hyper tuned model achieved 94% accuracy with a learning rate of 0.001. Each trail runs for 20 epochs and each epoch took 180 seconds. Time taken to run each trail by the hyper tuned CNN model is about 3600 seconds.

### 4.1. Error Analysis

The confusion matrix obtained by machine learning model SVM to classify the ECG images into 6 classes like Normal, LBBB, PAC, PVC, RBBB, and VF is represented in Table 7. The correctly classified number of images is presented in diagonal elements of the confusion matrix. Out of 2179 images of the Normal category, 1743 images are correctly classified into the Normal category and remaining images are misclassified into different categories like LBBB, PAC, PVC, RBBB, and VF. Out of 6825 test images, 5460 images are correctly classified by the SVM machine learning model and obtained the highest accuracy among all the machine learning models.

Table 8 represents the confusion matrix obtained by the Naïve Bayes machine learning model. Out of 2179 images of the Normal category, 1590 images are correctly classified into the Normal category and remaining images are misclassified into different categories like LBBB, PAC, PVC, RBBB, and VF. Out of 6825 test images, 4816 images are correctly classified and this model obtained an accuracy of 0.73.

The confusion matrix obtained by the Logistic Regression machine learning model to classify the ECG images into 6 classes like Normal, LBBB, PAC, PVC, RBBB, and VF is represented in Table 9. Out of 2179 images of the Normal category, 1525 images are correctly classified into the Normal category and remaining images are misclassified into different categories like LBBB, PAC, PVC, RBBB, and VF. Out of 6825 images, 4775 test images are correctly classified by the Logistic Regression model and obtained the accuracy of 0.70.

The confusion matrix obtained by the deep learning model CNN-Baseline model to classify the ECG images into 6 classes like Normal, LBBB, PAC, PVC, RBBB, and VF is represented in Table 10. Out of 2179 images of the Normal category, 1982 images are correctly classified into the Normal category and remaining images are misclassified into different categories like LBBB, PAC, PVC, RBBB, and VF. The developed CNN-Baseline model classifies 6005 images correctly out of 6825 images and obtained an accuracy of 0.91.

The confusion matrix obtained by deep learning model CNN-Hyper-tuned model to classify the ECG images into 6 classes like Normal, LBBB, PAC, PVC, RBBB, and VF is represented in Table 11. Out of 2179 images of the Normal category, 2048 images are correctly classified into the Normal category and remaining images are misclassified into different categories like LBBB, PAC, PVC, RBBB, and VF. Out of 6825 images, the proposed novel CNN-hyper tuned model correctly classifies 6413 images correctly and obtained an accuracy of 0.94.

## 5. Conclusion

This research work concentrates on developing an ECG-based image classification system that can be used to classify arrhythmia into different categories such as Normal, LBBB, PAC, PVC, RBBB, and VF using machine learning and deep learning models. ECG image-based heartbeat dataset collected from Kaggle and UCI repository is used for an analysis purpose. Initially, the data augmentation technique is used to enlarge the dataset. Then, machine learning models like Support Vector Machine, Naïve Bayes, and Logistic Regression are used for diagnosis. In order to extract high level features and to provide improved performance over machine learning algorithms, this research work utilizes deep learning-based Convolutional Neural Network approach called the CNN-Baseline model for arrhythmia detection. Further, to obtain optimal combination of parameters that minimizes loss function and produces better result in CNN, hyperparameter tuning is adopted in CNN and the CNN-Hyper-tuned model is developed. The proposed system utilizes the hyper-tuned model that employs Keras tuner to optimize hyperparameters used in the CNN-Baseline model. The result shows that the CNN-Hyper-tuned model applied on augmented dataset outperforms than other machine learning models and the CNN-Baseline model with 94% accuracy. Both machine learning and deep learning algorithms require long processing time and expensive also. In the future, transfer learning techniques like pretrained models will be utilized for classifying arrhythmia types.

## Figures and Tables

**Figure 1:** The proposed system work flow.

**Figure 2:** Shape of ECG images with different arrhythmia types.

**Figure 3:** Sample augmented ECG image.

**Figure 4:** Convolutional neural network-baseline model.

**Figure 5:** Hyperparameter tuning process workflow.

**Figure 6:** Hyper tuned Model Work Flow.

**Figure 7:** Performance evaluation of proposed models based on precision.

**Figure 8:** Performance evaluation of proposed models based on recall.

**Figure 9:** Performance evaluation of proposed models based on F1-Score.

**Figure 10:** Performance evaluation of proposed models based on F1-Score.

**Figure 11:** Accuracy and loss values of CNN-Baseline model.

**Table 1:** Literature study.

Author	Model	Approach	Dataset	Evaluation
Acharya et al. [12]	Convolutional Neural Network	Deep CNN with 11 input layers and 4 output neurons	MIT-BIH	Accuracy—92.5%
Isin and Ozdalili [13]	Artificial Neural Network and transferred deep learning	Transferred deep CNN is used to extract features and then applied Artificial Neural Network (ANN)	MIT-BIH	Accuracy—92%
Zubair et al. [14]	Convolutional Neural Network and LSTM	Dropout regularization	MIT-BIH	Accuracy—91.8% Appl. Sci. 9, 14 (2019), 2921. DOI: 10.3390/app9142921
Ribeiro et al. [15]	Deep Neural Network	Stacked transformations	CODE	F1-Score—above 80%
Porumb et al. [16]	CNN	Multilayer perceptron for raw signal classification	MIT-BIH(250 samples)	Accuracy—97%
Khan et al. [17]	Deep Neural Network	MobileNet	Manual dataset	Accuracy—98%
Atal and Singh [18]	Deep CNN	Bat-Rider Optimization algorithm	MIT-BIH	Accuracy—93.19%
Zheng et al. [19]	Ensemble models	Hyper-tuned classification model	Manually generate dataset	F1-Score—97%
Mathunjwa et al. [20]	CNN	Hyperparameter tuning	MIT-BIH	Accuracy—95. 3%
Jun et al. [21]	CNN	AlexNet, VGGNet	MIT-BIH	Accuracy—99.05%
Hu et al. [7]	CNN-Transformer-based model	Classification and positioning	MIT-BIH	Accuracy—99.49%
Yıldırım et al. [22]	1D-CNN	ECG signal fragments based on one lead	MIT-BIH	Accuracy—91.33%
Li et al. [23]	SE-ResNet deep learning model	19-layer deep squeeze-and-excitation residual network	MIT-BIH	Accuracy—99.61%
Sharma et al. [10]	LSTM	Rhythm-based method	MIT-BIH	Accuracy—90.07%
Simonyan and Zisserman [24]	Deep learning	ConvNet	ILSVRC-2012	Accuracy—93.2%
Damaševičius et al. [25]	Machine learning	KNN	Time series dataset	Accuracy—86%
Naz et al. [26]	Deep learning	AlexNet, VGG-16, Inception-V3	MIT-BIH	Accuracy—97.6%

**Table 2:** Augmented ECG image dataset.

Class labels	Training data	Test data
Normal	7346	2179
LBBB	504	341
PAC	2054	1503
PVC	2759	1645
RBBB	2239	915
VF	439	242

**Table 3:** CNN-Baseline model summary.

Layer (type)	Output shape	Number of parameters
conv2d (Conv2D)	(None, 62, 62, 32)	320
max_pooling2d (MaxPooling2D)	(None, 31, 31, 32)	0
Flatten (flatten)	(None, 30752)	0
Dense (dense)	(None, 128)	3,936,384
Dense_1 (dense)	(None, 6)	774
Total params: 3,937,478	Trainable params: 3,937,478	Nontrainable params: 0

**Table 4:** CNN-Hyper-tuned model summary.

Layer (type)	Output shape	Number of parameters
Conv2d_4 (Conv2D)	(None, 62, 62, 16)	448
Conv2d_5 (Conv2D)	(None, 60, 60, 16)	2320
Max_pooling2d_2 (MaxPooling 2D)	(None, 15, 15, 16)	0
Dropout (dropout)	(None, 15, 15, 16)	0
Conv2d_6 (Conv2D)	(None, 13, 13, 32)	4640
Conv2d_7 (Conv2D)	(None, 11, 11, 64)	18496
Max_pooling2d_3 (MaxPooling 2D)	(None, 5, 5, 64)	0
Dropout (dropout)	(None, 5, 5, 64)	0
Flatten_1 (flatten)	(None, 1600)	0
Dense_3 (dense)	(None, 128)	204928
Dropout_2 (dropout)	(None, 128)	0
Dense_3 (dense)	(None, 6)	774
Total params: 231,606	Trainable params: 231,606	Nontrainable params: 0

**Table 5:** Performance evaluation.

Model	Precision	Recall	F1-Score	Accuracy
SVM	0.84	0.75	0.79	0.80
Naïve Bayes	0.77	0.79	0.78	0.73
Logistic Regression	0.67	0.80	0.73	0.70
CNN-Baseline model	0.88	0.90	0.89	0.91
CNN-Hyper-tuned model	0.92	0.90	0.91	0.94

**Table 6:** Hyperparameters and their values in the CNN-Hyper-tuned model.

Hyperparameters	Trail 1	Trail 2	Trail 3	Trail 4	Trail 5
conv_1_filter	80	80	112	96	64
conv_1_kernel	5	5	5	3	3
conv_2_filter	56	64	56	64	48
conv_4_filter	32	40	48	48	56
dense_1_units	80	80	128	64	64
dense_2_units	80	96	64	112	128
Learning_rate	0.01	0.001	0.01	0.001	0.01
Score	0.78123	0.83211	0.88993	0.94375	0.93531

**Table 7:** Confusion matrix–SVM.

	Normal	LBBB	PAC	PVC	RBBB	VF
Normal	1743	101	102	105	107	71
LBBB	11	273	17	15	11	14
PAC	52	218	1316	34	15	10
PVC	63	41	47	1202	106	44
RBBB	45	30	28	40	732	40
VF	9	15	7	10	7	194

**Table 8:** Confusion matrix–Naïve Bayes.

	Normal	LBBB	PAC	PVC	RBBB	VF
Normal	1590	182	101	93	113	100
LBBB	23	249	16	15	17	21
PAC	120	117	1200	98	63	47
PVC	56	153	76	1097	42	79
RBBB	23	39	87	44	667	55
VF	10	17	15	11	13	176

**Table 9:** Confusion matrix–Logistic Regression.

	Normal	LBBB	PAC	PVC	RBBB	VF
Normal	1525	203	63	159	178	51
LBBB	13	238	35	16	10	29
PAC	56	189	1151	83	153	13
PVC	51	73	67	1052	203	57
RBBB	98	58	23	62	640	34
VF	19	23	12	10	9	169

**Table 10:** Confusion matrix–CNN-Baseline model.

	Normal	LBBB	PAC	PVC	RBBB	VF
Normal	1982	18	46	52	63	18
LBBB	11	310	9	5	2	4
PAC	75	21	1496	11	26	16
PVC	13	25	34	1367	42	22
RBBB	13	11	19	23	832	12
VF	1982	18	46	52	63	18

**Table 11:** Confusion matrix–CNN-Hyper-tuned model.

	Normal	LBBB	PAC	PVC	RBBB	VF
Normal	2048	29	15	43	23	21
LBBB	1	320	3	4	2	11
PAC	26	14	1546	16	28	15
PVC	11	13	35	1412	25	7
RBBB	9	11	12	10	860	13
VF	2	1	3	4	5	227

## Data Availability

The data used to support the findings of this study are included within the article.
